# Effects and Mechanism of Zishen Jiangtang Pill on Diabetic Osteoporosis Rats Based on Proteomic Analysis

**DOI:** 10.1155/2021/7383062

**Published:** 2021-09-24

**Authors:** Shufang Chu, Deliang Liu, Hengxia Zhao, Mumin Shao, Xuemei Liu, Xin Qu, Zengying Li, Jinhua Li, Huilin Li

**Affiliations:** ^1^Department of Endocrinology, Shenzhen TCM Hospital, The Fourth Clinical Medical College of Guangzhou University of Chinese Medicine, Shenzhen 518033, China; ^2^Department of Pathology, Shenzhen TCM Hospital, The Fourth Clinical Medical College of Guangzhou University of Chinese Medicine, Shenzhen 518033, China

## Abstract

**Objective:**

To explore the effect and mechanism of ZJP on DOP rats by proteomic analysis.

**Materials and Methods:**

After the establishment of diabetes model by Streptozocin (STZ, 60 mg/kg), 40 Wistar rats were equally divided into normal group, model group (diabetic rats), high-dose group (3.0 g/kg/d ZJP), and low-dose group (1.5 g/kg/d ZJP) and received treatment for 3 months. Histological changes in bone and pancreas tissues were observed by hematoxylin and eosin staining, electron microscopy, and immunofluorescence. Proteomic and bioinformatic analyses were performed to identify the differentially expressed proteins. The fingerprint and active ingredients of ZJP were identified via high-performance liquid chromatography (HPLC).

**Results:**

Compared with the model group, ZJP could rescue the weight, fasting blood glucose, and fasting insulin of rats in both high-dose and low-dose group. ZJP could also improve the microstructures of pancreatic islet cells, bone mass, and trabecular and marrow cavities in DOP rats. Bioinformatic analysis suggested that ZJP might influence DOP via multiple pathways, mainly including ribosomes, vitamin digestion and absorption, and fat digestion and absorption. The primary active ingredients, including notoginsenoside R1, ginsenoside Rg1, ginsenoside Re, icariin, and ginsenoside Rb1, were detected.

**Conclusion:**

ZJP could significantly improve the histomorphology and ultrastructure of bone and islets tissues and might serve as an effective alternative medicine for the treatment of DOP.

## 1. Background

DOP is a common diabetic complication [1, 2]. The main pathological changes associated with DOP are a decrease in bone mass per unit volume, a reduction in bone strength, and an increase in bone fragility [3, 4]. With the aging of the global population, the incidence of DM is increasing every year, which directly leads to an increase in the incidence of DOP [5, 6]. At present, the treatment of DOP is mainly based on antiosteoporosis drugs [7, 8]. Western medicine treatments generally include taking calcium, vitamin D, sex hormones, bisphosphonates, calcitonin, and/or fluoride or using monoclonal antibodies [9–11]. However, the therapeutic effects of such drugs are still controversial, and some patients cannot tolerate their side effects or afford their expensive prices. As such, there is an urgent need to identify the mechanism of osteoporosis in patients with diabetes in an effort to identify more cost-effective treatments.

Recently, a large number of experimental and clinical studies detailing the treatment of DOP have affirmed the efficacy of Traditional Chinese Medicine (TCM) [12–14]. Zishen Jiangtang Pill (ZJP) is a TCM compound developed by Shenzhen TCM Hospital. The components of ZJP have the functions of nourishing the breath feminine, nourishing the kidneys, and strengthening the bones. Its use is in line with the theory of “kidney dominating bone” for the treatment of osteoporosis. A previous study has found that ZJP has a positive function with regard to hypoglycemic action, decreasing lipids, and improving insulin sensitivity and revealed that ZJP could play an antiosteoporosis role on multiple targets, as based on *in vitro* experiments [15]. However, the molecular mechanism by which ZJP works is still not fully understood.

Based on a previous study, we have known that ZJP has glycemic control effects with regulating effects on bone metabolism and hypothesized that ZJP can effectively treat DOP rats. In order to explore the effect and mechanism of ZJP on diabetic osteoporosis rats, we established a DOP rat model and treated these rats with different doses of ZJP and observed the bones and histomorphology of pancreatic tissue. By using gene ontology (GO) and Kyoto Encyclopedia of Genes and Genomes (KEGG) analysis, these results reveal that ZJP may affect DOP via multiple pathways.

## 2. Materials and Methods

### 2.1. Drugs, Reagents, and Antibodies

Zishen Jiangtang Pills (ZJP) were prepared by the Pharmacy Department of Shenzhen TCM Hospital. The main components were *Astragali Radix, Rehmanniae Radix Praeparata, Epimedii Folium, Notoginseng Radix et Rhizoma, Codonopsis Radix, Achyranthis Bidentatae Radix, Schisandrae Chinensis Fructus, Polygonati Rhizoma,* and *Drynariae Rhizoma* (Batch No. Guangdong Z20070085). The specific formula composition and preparation method are referred from chen et al [16].

The main reagents and antibodies used are as follows: STZ and carboxymethyl cellulose sodium (CMC) (No. S0130/C4888, Sigma, USA), insulin primary antibody (No. 3014s, CST, USA), fluorescent secondary antibody (No. 111-585-003, Jackson ImmunoResearch Laboratories, Inc., USA; and No. A23210, Abbkine, USA), glucagon primary antibody (No. ab10988, Abcam, UK), DAPI fluorescent seal tablets (No. 0100-20, Southern Biotech), chromatographically pure acetonitrile (Merck, USA), and the reference products including notoginsenoside R1, ginsenoside Rg1, ginsenoside Re, icariin, and ginsenoside Rb1 (China Food and Drug Testing Institute). ZJP is evenly mixed and suspended in CMC.

### 2.2. Animals

A total of 70 2-month-old Specific Pathogen-Free (SPF) male Wistar rats, weighing from 160 to 190 g, were purchased from the experimental animal center of Southern Medical University with a quality certificate No. 44002100006561. The animals were housed in the SPF room in Shenzhen Municipal Center for Disease Control and Prevention, with an ambient temperature of 18–22 °C, natural circadian rhythm illumination (12 h: 12 h), and environmental humidity of 40–70%. The rats were kept in microisolator cages and were given free access to food and water. All animal experiments were in accordance with the Animal Research Ethics Committee and approved by the Animal Protection and Use Committee of the Guangdong Experimental Animal Center (approval number: IACUC-G16003).

### 2.3. Plasma Measurements

Blood samples were collected from the animals' tail veins. The fasting blood glucose (FBG) levels and fasting plasma insulin (FINS) were determined by test assay kits abiding by the manufacturer's instructions (Roche Diagnostics Co., Ltd., Germany, and USBiological Co., Ltd., United States).

### 2.4. Bone Mineral Density (BMD) Detection

The BMD of lumbar vertebrae (L1–L4) was detected by using dual-energy X-ray absorptiometry (DEXA) scanning system (GE, United States) on the last day of the experiment. The measurement parameters are dual-energy voltage 41 kVp and 100 kVp, scanning window width 18 am, and scanning rate 4.8 s/am.

### 2.5. Establishment of a Rat Diabetes Model

Rats were adaptively fed for 2 weeks, and 10 rats were randomly selected as normal controls. The remaining 60 rats were used to establish the diabetes model. After fasting for 12 h, rats were injected intraperitoneally with 0.2% STZ (diluent 0.1 M citrate-sodium buffer, pH 4.5) at a dose of 60 mg/kg [17]. The blood glucose of the rats was measured using a blood glucose meter 72 h after administration. Rats with a fasting blood glucose >16.7 mmol/L were fed commonly for 2 weeks. Those rats that still had a fasting blood glucose >16.7 mmol/L were considered as successful models [18]. The normal control group was injected intraperitoneally with the same amount of 0.1 M citrate-sodium buffer (pH = 4.5). In the diabetes induction, 8 animals were dead and 12 animals were failed. The failed animal studies were performed under isoflurane anesthesia and every effort was made to minimize suffering. Finally, a total of four groups with 10 rats in each group were obtained. The rats of four groups then received treatment for 3 months. The normal group and model group were given 0.5% sodium carboxymethyl cellulose 10 mL/kg/day via intragastric administration, and the high-dose (3.0 g/kg/d ZJP) and low-dose (1.5 g/kg/d ZJP) groups were simultaneously given 0.5% sodium carboxymethyl cellulose 10 mL/kg/day via intragastric administration. At the end of the treatment, all of the rats were fasted for 12 h and then anesthetized using sodium pentobarbital (50 mg/kg) and sacrificed via abdominal aorta bleeding. The blood was obtained, and the pancreas and bone tissues were stored at -80 °C. After muscle and tendons were removed, the femoral bone was utilized for biochemical and histologic evaluation.

### 2.6. Hematoxylin and Eosin (H&E) Staining

Pancreatic tissues were sliced, fixed in 4% paraformaldehyde, rinsed with water for 24 h, dehydrated with an ethanol gradient, placed in anhydrous acetone, and embedded in polymethyl methacrylate [19]. H&E staining was performed as follows: xylene for 5 min, xylene for 3 min, 100% alcohol for 30 s, 100% alcohol for 30 s, 95% alcohol for 30 s, 90% alcohol for 30 s, hematoxylin staining for 10–15 min, 1% hydrochloric acid alcohol differentiated slice for 10 s, 1% eosin staining for 3 min, 90% alcohol for 30 s, 95% alcohol for 30 s (2x), 100% alcohol for 30 s (3x), carbonic acid xylene for 30 s, xylene for 30 s (3x), and a neutral gum seal.

### 2.7. Double-Label Pancreatic Immunofluorescence

The paraffin slices were baked at 60°C, dewaxed with xylene and ethanol, and repaired using citrate antigen repair solution. The slices were then incubated with insulin (1 : 400) and glucagon (1 : 1000) primary antibodies in the dark at 4°C overnight. The slices were then incubated with a fluorescent secondary antibody (1 : 100) at 37°C in the dark for 1 h, stained with DAPI, and sealed using a fluorescent sealing tablet. The positive islet beta cells appeared red, the positive islet alpha cells appeared green, and the nuclei appeared blue.

### 2.8. Pancreatic Transmission Electron Microscopy

Pancreatic tissues were fixed with 2.5% glutaraldehyde, dehydrated in ethanol, penetrated with propylene oxide, and embedded with a 1 : 1 propylene oxide and resin mixture for 2 h, pure resin for 2 h, and resin at 48 °C for 10 h. The samples were then sliced at 500–1000 nm, stained with toluidine blue, sliced at 70 nm, and stained with lead and uranium.

### 2.9. Femoral Electron Microscope Scanning

The fixed bone tissue sections were processed as follows: sections were stained with Weigert's iron lignin on a glass slide for 40 min and rinsed with water until it turned blue. These were then incubated in 1% hydrochloric acid ethanol and washed with water until it turned blue, dyed with Van Gieson picric acid-magenta solution for 3 min, dehydrated with 95% ethanol and anhydrous ethanol, quickly dipped in fresh anhydrous ethanol, and then blotted dry. After the above treatment, the sections were immersed in an acetonitrile solution, which was then replaced with 70%, 80%, 90%, 95%, and 100% acetonitrile, soaked for 15–20 min each time, and finally replaced with 100% acetonitrile and dried. The sections were then sprayed with carbon and gold and observed under an electron microscope.

### 2.10. Proteomic Analysis

The proteins were extracted from the rats' bone tissues in different groups. The extracted protein samples were subjected to reductive alkylation treatment to open the disulfide bonds for subsequent enzymatic hydrolysis of the proteins. Trypsin and 8-plex iTRAQ reagent (AB Sciex, Cat. No. 4381664) were used to label the protein. The mixed peptides were preisolated using high pH reverse phase chromatography, and liquid chromatography was performed coupled with tandem mass spectrometry (LC-MS/MS) analysis. The mass spectrometry data was assessed using Protein Pilot software (AB, Version 5.0) and aligned for identification; the database used was UniProtKB/Swiss-Prot. The identification criteria for the differentially expressed proteins had a fold difference of ≥1.5 or ≤0.667, and the number of unique peptides per protein ≥2 and <0.05 was considered to be a significant difference.

The OmicsBean (https://www.omicsbean.cn/) multifunctional bioinformatics analysis tool, integrated STRING (https://www.string-db.org) biological database, and Cytoscape software were used to perform enrichment analysis on the identified differentially expressed proteins based on GO biological process, cellular component, and molecular function. Additionally, KEGG (https://www.kegg.jp/kegg/pathway.html) biological pathway enrichment analysis was performed on the differentially expressed proteins.

### 2.11. HPLC Fingerprinting and Active Ingredient Detection

A reference solution that contained notoginsenoside R1, ginsenoside Rg1, ginsenoside Re, icariin, and ginsenoside Rb1 was mixed with methanol at a concentration of 0.1 mg/mL. The ZJP powder was dissolved in 100% methanol and filtered as test solution. The reference solution and the test solution were tested via HPLC, and the characteristic maps of both solutions were obtained. The chromatographic conditions were as follows: octadecyl silane-bonded silica gel was used as filler, and gradient elution was carried out at a detection wavelength of 203 nm. The column was an Agilent TC-C18 (250 mm × 4.6 mm, 5 *μ*m) with water as mobile phase A and acetonitrile as mobile phase B (gradient elution: 0–12 min, 81% A, and 12–60 min, 81%–64% A; flow rate 1.0 mL/min; and a detection wavelength of 203 nm).

### 2.12. Statistical Analysis

The obtained data were statistically analyzed and processed using State 12.0 software, and the measured data were expressed as the mean ± standard deviation ($\bar{x}\pm \text{SD}$). One-way analysis of variance (ANOVA) was used to assess the differences between the groups, and the Bonferroni test was used for multiple comparisons between the groups. Wilcoxon rank-sum test was used for comparison between the group data which did not conform to a normal distribution or variance. Statistical significance was defined as *P* < 0.05.

## 3. Results

### 3.1. Body Weight, Fasting Blood Glucose, and Fasting Insulins

The body weight of the model group (238.7 ± 22.08 g) was significantly lower than that in the normal group (408.8 ± 21.06 g) (*P* < 0.01). Compared with the model group, the rats in the high-dose ZJP group (308.3 ± 19.35 g) and the low-dose ZJP group (305.9 ± 13.25 g) had gained significant weight (*P* < 0.01). The results are shown in Figure 1(a). In addition, as shown in Figure 1(b), both the high-dose (13.16 ± 2.15 mM) and low-dose groups (14.66 ± 1.22 mM) of ZJP could effectively reduce the fasting blood glucose of the model group (23.79 ± 5.54 mM) (*P* < 0.01), and there was no significant difference between the two groups. Also, ZJP could significantly improve the fasting insulin of model group (514.0 ± 180.7 pg/mL) (*P* < 0.01), while there was no significant difference between high-dose (2360 ± 718.2 pg/mL) and low-dose groups (2508 ± 925 pg/mL) (Figure 1(c)).

### 3.2. ZJP Can Improve the BMD of Lumbar Vertebrae in DOP Model Rats

As shown in Figure 1(d), the BMD of the model group (0.11 ± 0.01 g/cm^2^) was significantly lower than that in the normal group (0.16 ± 0.01 g/cm^2^) (*P* < 0.001). Compared with the model group, the rats in the high-dose ZJP (0.12 ± 0.01 g/cm^2^) and the low-dose ZJP groups (0.13 ± 0.01 g/cm^2^) had proven the BMD of lumbar vertebrae in DOP model rats (*P* < 0.001 and *P* < 0.05, respectively.).

### 3.3. ZJP Can Improve the Status of Pancreatic Islet Cells in DOP Model Rats

We assessed the effect of ZJP on pancreatic islet cells by H&E staining, immunofluorescence, and transmission electron microscopy. The islet cells in the normal group were lightly stained, with a high cell density, uniform distribution, and regular morphology (Figures 2(a) and 2(e)). The mitochondria, endoplasmic reticulum, and Golgi were abundant in the cytoplasm of the normal group (Figure 2(i)). In the model group, the islets were significantly reduced, their shape was irregular, their cell density was reduced, and more cells presented with nuclear pyknosis. The peripheral acinar cells also demonstrated substantial atrophy and degeneration (Figures 2(b) and 2(f)). Moreover, the number of mitochondria was decreased, and they were swollen and deformed, the endoplasmic reticulum had expanded to different extents, and a degranulation phenomenon could be seen (Figure 2(j)). The pancreatic islet structures in the high-dose and low-dose ZJP groups were significantly improved compared with the model group. In these treatment groups, the islet size was basically normal, the morphology was regular, the islet cells were arranged neatly, the density was acceptable, and the numbers of atrophied and degenerated islet cells were decreased (Figures 2(c), 2(d), 2(g), and 2(h)). Additionally, in these treatment groups, the endoplasmic reticulum was not significantly expanded (Figures 2(k) and 2(l)).

### 3.4. ZJP Can Improve the Histological Morphology of Bone Tissues in DOP Model Rats

In addition to the effects of bone mass reduction, DOP is also related to bone structure factors and the number of microinjuries in the bone [20, 21]. Therefore, we performed electron microscopy to assess for these changes in the bone microstructures. The bone density of the femurs in the normal group was thick and the trabecular bones were arranged neatly. The surface of the trabecular bone was regular and smooth, the gap between the trabeculae was small, and the collagen fibers were neatly arranged in the trabecular bone (Figure 3(a)). In the model group, the bone density appeared to be significantly thinner, the marrow cavity was larger, the trabecular bone connection was interrupted, and the reticular structure was destroyed (Figure 3(b)). The trabecular bone structures in the high-dose and low-dose ZJP groups were more organized compared with the model group. The bone marrow cavities were also smaller (Figures 3(c) and 3(d)).

### 3.5. GO and KEGG Analysis of ZJP Function in DOP Model Rats

In order to better clarify how ZJP exerts its antiosteoporosis function, we carried out proteomic GO and KEGG analyses. We classified the altered proteins after low-dose ZJP treatment into GO classification due to the equal effect with high-dose ZJP treatment on DOP rats. Compared to the normal group, the results in the model group indicated that DOP mostly resulted in protein changes in biological process including anatomical structure development (13%), response to stress (13%), biosynthetic process (12%), and cellular nitrogen compound metabolic process (12%) (Figure 4(a)). The molecular functions of these proteins most likely reflected ion binding (19%), RNA binding (17%), and enzyme binding (15%) (Figure 4(b)). As for the cellular component, the highest probability of existence included the extracellular region (17%), organelle (17%), and cytoplasm (16%) (Figure 4(c)). By comparing the low-dose ZJP group with the model group, we arrived at a similar conclusion with regard to these three categories (Figures 4(d)–4(f)).

We then performed pathway enrichment analysis on the differentially expressed proteins. Comparing the normal group with the model group, the pathways with the highest degree of enrichment involved the following aspects: fatty acid elongation, arginine and proline metabolism, fatty acid degradation, PPAR signaling pathway, fat digestion and absorption, adipocytokine signaling pathway, and DNA replication (Figure 5(a)). Meanwhile, comparing the model group with ZJP treatment groups, the most enriched pathways were ribosome, vitamin digestion and absorption, DNA replication, arginine and proline metabolism, and fat digestion and absorption (Figure 5(b)).

### 3.6. ZJP Fingerprint and Active Ingredients

We first determined the fingerprint map of ZJP via HPLC and identified its active ingredients (Figure 6). There were five major characteristic peaks in the map with relative retention time specifications, including notoginsenoside R1 (peak 1), ginsenoside Rg1 (peak 2), ginsenoside Re (peak 3), icariin (peak 4), and ginsenoside Rb1 (peak 5).

## 4. Discussion

DOP is a common complication of DM. With the aging of the global population, the incidence of both DM and DOP is becoming higher and is affecting people's quality of life. At present, the treatment for DOP includes three types: supplementation of calcium and vitamin D [22, 23], inhibition of bone resorption with drugs such as bisphosphonates [24–26], and promotion of bone formation with drugs such as PTH1-34 [27, 28]. However, the overall effect of these treatments is not particularly good, with a high rate of side effects and a high cost. Currently, numerous studies are focusing on the effects of TCM with regard to osteoporosis [29–31], but the concise role and mechanism underlying such treatments are still unclear. As such, it is important to understand the molecular mechanism and related pathogenesis of DOP, so as to help identify an effective therapy. This study found that ZJP can significantly improve the BMD of lumbar vertebrae in DOP model rats, the histomorphology, and ultrastructure of bone and pancreatic islet tissues. After further proteomic analysis of differentially expressed proteins, it is found that ZJP can exert its effects by affecting various aspects of glucose metabolism and bone metabolism. The influence of DOP, which involves multiple pathways, indicates that ZJP, a traditional Chinese medicine compound, plays a role through the characteristics of multiple components and multiple targets and may be used as an effective alternative drug for the treatment of DOP.

A previous study has demonstrated that ZJP can effectively improve glucose metabolism and abnormal bone metabolism and regulate blood and urinary metabolism in DOP rats [15]. ZJP has a clear hypoglycemic and lipid-lowering effect and can improve insulin sensitivity, promote resistance to oxidation, protect the vascular endothelium, and reduce the level of inflammatory factors [32, 33]. Based on the establishment of our DOP rat model, we found that ZJP could reduce the weight loss of rat caused by DOP and improve the fasting blood glucose and fasting insulin of these rats (Figure 1). The most important changes occurring in patients with DOP involve alterations in blood glucose and the skeletal system. Therefore, microscopic analyses of islet cells and bone tissues were performed in the present study. The results indicated that ZJP conferred an obvious improvement to the histomorphology and ultrastructure of islets (Figure 2) and could improve bone formation, reduce bone resorption, increase bone density, and improve the bone microstructure (Figure 3). These pathology results support our previous findings [15] that ZJP was shown to exert its influence by affecting aspects of glucose metabolism and bone metabolism.

To further investigate the potential mechanism of ZJP in the treatment of DOP, we performed proteomic GO and KEGG analyses on the identified differentially expressed proteins. The results revealed that ZJP most likely affected ion binding, RNA binding, and enzyme binding involved in several biological processes, including anatomical structure development, response to stress, biosynthetic processes, and cellular nitrogen compound metabolic processes. The roles of ZJP in these aspects are closely related to known factors related to the occurrence and development of DOP. Moreover, these roles are reflected in several aspects of DOP, such as bone structure changes and blood metabolism. The highest probabilities of existence with regard to the cellular component were the extracellular region, organelles, and cytoplasm, indicating that it is possible that ZJP might have some functions affecting the cellular microenvironment. The enrichment pathways identified mostly referred to the ribosome, vitamin digestion and absorption, DNA replication, arginine and proline metabolism, and fat digestion and absorption, indicating that ZJP is closely related to changes in body weight and calcium absorption as well as protein synthesis. However, to further characterize the protein signaling network associated with the treatment of DOP via ZJP, it will be necessary to further identify the specific target genes via additional methods, both *in vitro* and *in vivo*, in an effort to define the mechanism of action of ZJP with regard to the treatment of DOP.

ZJP is a Chinese herbal compound developed by Shenzhen TCM Hospital, and this study was the first to define the fingerprint map of ZJP via HPLC and ascertain the primary active ingredients, including notoginsenoside R1, ginsenosideRg1, ginsenoside Re, icariin, and ginsenoside Rb1. Thus, notoginsenoside R1, ginsenoside Rg1, ginsenoside Re, icariin, and ginsenoside Rb1 together were found to have both an antihypoglycemic action and an antiosteoporosis effect in the previous study [34, 35]. Pharmacological studies have confirmed that epimedium extracts can inhibit the activity of osteoclasts via various means and promote the differentiation of osteoblasts and increased bone formation and bone density [36–38]. Ginsenoside Rg1 treatment of diabetic rats was associated with reduced oxidative stress and attenuated myocardial apoptosis [35]. Icariin could significantly regulate the nNOS and calponin in penile tissues of all rats [34]. Icariin attenuates titanium-particle inhibition of bone formation by activating the Wnt/*β*-catenin signaling pathway *in vivo* and *in vitro* [37]. These observations provided theoretical support for the prevention and treatment of DOP by ZJP.

## 5. Conclusions

Overall, this study identified the main active components of ZJP and determined that ZJP could significantly improve the histomorphology and ultrastructure of bone and islets tissues using a DOP rat model and might serve as an effective alternative medicine for the treatment of DOP. In the further study, we will focus on one compound as a representative ingredient and verify the predicted mechanisms.

## Figures and Tables

**Figure 1:** Body weight. (a) Fasting blood glucose and (b) and fasting insulin (c) of each group. (d) BMD.

**Figure 2:** Pancreatic microstructure in each group. (a–d) H&E staining (×400); (e–h) insulin-glucagon double-label immunofluorescence (×400); (i–l) transmission electron microscopy (×5000). A, E, and I: normal group. B, F, and J: model group. C, G, and K: high-dose ZJP group. D, H, and L: low-dose ZJP group.

**Figure 3:** Scanning electron micrograph of a femur from each group (×100). (a) Normal group. (b) Model group. (c) High-dose ZJP group. (d) Low-dose ZJP group.

**Figure 4:** GO analysis results for the different groups of DOP rats. The normal group versus model group: (a) biological process, mainly differenced in response to stress, anatomical structure development, and biosynthetic process; (b) molecular function, mainly differenced in ion binding, RNA binding, and enzyme binding; (c) cellular component, mainly differenced in the extracellular region, organelle, and cytoplasm. The model group versus low-dose ZJP group: (d) biological process, mainly differenced in anatomical structure development, biosynthetic process, and cellular nitrogen compound metabolic process; (e) molecular function, mainly differenced in ion binding, enzyme binding, and RNA binding; (f) cellular component, mainly differenced in the cytoplasm, extracellular region, and organelle.

**Figure 5:** Pathway analysis of the differentially expressed proteins between the different groups. (a) Normal group versus model group, mainly in fatty acid elongation, arginine and proline metabolism, and fatty acid degradation pathway. (b) Model group versus low-dose ZJP group, mainly in ribosome, vitamin digestion and absorption, and DNA replication pathway.

**Figure 6:** HPLC fingerprint of ZJP. Peak 1: notoginsenoside R1; peak 2: ginsenoside Rg1; peak 3: ginsenoside Re; peak 4: icariin; peak 5: ginsenoside Rb1.

## Data Availability

All the data and materials of this manuscript are available.
